The article "Effusive-Constrictive Pericarditis in a Young Active Duty Male" was published in 2020. Journal: Cureus.

# Effusive-Constrictive Pericarditis in a Young Active Duty Male

**DOI:** 10.7759/cureus.9997

**Published:** 2020-08-24

**Authors:** Arjun G Kalra, Alec J Sharp, Laith Dinkha, Rosco Gore

**Affiliations:** 1 Internal Medicine, Brooke Army Medical Center, Fort Sam Houston, USA; 2 Cardiology, Brooke Army Medical Center, Fort Sam Houston, USA

**Keywords:** tamponade, tte, malignancy, radiation, echocardiogram, ecp, hemodynamic instability, heart failure

## Abstract

Effusive-constrictive pericarditis (ECP) is a rare clinical entity resulting from accumulating pericardial fluid within a stiff, non-compliant pericardium. There are a number of etiologies for ECP, which include malignancy, radiation, post-surgical causes, infectious, and collagen disorders. Clinically, ECP often presents as right-sided heart failure, or in advanced cases, cardiac tamponade. Symptoms may persist despite treatment with pericardiocentesis, and may warrant consideration for pericardiectomy for more definitive management. Invasive hemodynamic evaluation with cardiac catheterization remains the gold standard for diagnosis of ECP; however, echocardiography can provide a definitive diagnosis with high sensitivity and specificity. Echocardiographic features suggestive of ECP include ventricular septal motion abnormalities, such as interdependence, accentuated longitudinal motion of the heart, and altered respirophasic ventricular filling. While these features have been well established and can lead to the diagnosis of ECP, they are rarely observed in clinical practice. We present a case of ECP in a 25-year-old active duty male with a history of chest wall myoepithelial carcinoma who clearly demonstrated such echocardiographic findings of ECP.

## Introduction

Pericardial effusions are a commonly observed finding on echocardiographic evaluation. The effusions can vary in size from trivial, defined as <50 mL, to large, defined as >500 mL of fluid contained within the pericardial space. While the size of the pericardial effusion may provide clues as to its underlying etiology, it often correlates poorly with its hemodynamic effects on the heart. Clinical presentation and patient symptoms may vary widely and can include chest pain, dyspnea, and/or hemodynamic instability if cardiac tamponade is present. In general, most pericardial effusions can be monitored with serial imaging, and do not require drainage with pericardiocentesis, but in symptomatic patients with moderate to large pericardial effusions, or in those with findings of cardiac tamponade, pericardiocentesis can be a life-saving intervention. Immediate improvement in the patient’s symptoms and clinical condition is typically observed. Therefore, persistent symptoms following pericardiocentesis should raise suspicion for the presence of effusive-constrictive pericarditis (ECP).

The article "Effusive-Constrictive Pericarditis in a Young Active Duty Male" was published in 2020. Journal: Cureus.

ECP is a rare clinical entity characterized by accumulating pericardial fluid within a stiff and non-compliant pericardium. Etiologies for ECP include malignancy-related conditions, radiation, post-surgical, infectious, or idiopathic [1-7]. Prevalence, while not fully known, is reported to range from 1% to 16% in patients presenting with pericarditis or cardiac tamponade [3,4]. Invasive hemodynamic evaluation with cardiac catheterization remains the gold standard for diagnosis; however, diagnosis can often be made by echocardiographic assessment following pericardiocentesis.

Herein, we report a case of an active duty soldier with a new pericardial effusion and clinical tamponade, who underwent pericardiocentesis and was found to have findings consistent with ECP on repeat echocardiographic evaluation.

## Case presentation

A 25-year-old non-smoking male with a history of chest wall myoepithelial carcinoma status post excision, chemotherapy, and radiation therapy with relapse in and progression of disease on pembrolizumab presents to the emergency department (ED) with 10 days of progressive dyspnea on exertion, palpitations, and 45-pound weight loss over the past three months. 

Initial evaluation consisted of a chest x-ray and CT of the chest with contrast, which revealed metastatic spread to the patient’s lungs including spread to the epicardium, and a new pericardial effusion (Figures 1, 2).

**Figure 1:** Chest X-ray showing enlarged cardiac silhouette (red arrow) as well as right hemithorax status post chest wall resection with remnant neoplastic process (white arrow)

**Figure 2:** CT findings representing metastatic foci of disease to lung and epicardium (white arrows) as well as pericardial effusion (red arrows) with coronal view (A) and transverse view (B)

Diagnostic transthoracic echocardiogram was then performed, which showed a very large circumferential pericardial effusion, measuring up to 4 cm along the right ventricular free wall, with associated findings concerning for tamponade physiology (Figure 3). 

**Figure 3:** Demonstration of pericardial effusion with respirophasic interventricular septal shifting Two-dimensional parasternal long-axis (A) demonstrating increased pericardial thickness (yellow arrowheads) and a moderate pericardial effusion (white asterisk) following pericardiocentesis. M-mode echocardiography (B) depicting ventricular septal shift towards the left ventricle (downward arrow) during inspiration and towards the right ventricle (upward arrow) during expiration. Simultaneous respirometric recording is shown at the bottom of the figures (green line). Two-dimensional parasternal short axis (C) showing a moderate circumferential pericardial effusion (white asterisk). M-mode echocardiography (D) depicting ventricular septal shift towards the right ventricle (upward arrow) during expiration and towards the left ventricle (downward arrow) during inspiration.

The article "Effusive-Constrictive Pericarditis in a Young Active Duty Male" was published in 2020. Journal: Cureus.

Urgent fluoroscopic-guided pericardiocentesis was then performed, removing 590 mL of serosanguinous fluid. A pigtail catheter drain was left in place for residual effusion, and subsequent serial echocardiography was performed, revealing a persistent small-to-moderate sized pericardial effusion with continued respirophasic septal shifting, and annulus reversus on tissue Doppler imaging suggestive for ECP as the underlying cause for this clinical presentation (Figures 3-5). 

**Figure 4:** Demonstration of constrictive pathophysiology via tricuspid and mitral inflow velocities with respiratory variation Pulse-wave Doppler findings from the tricuspid (A) and mitral (B) inflow velocities with simultaneous respirometric recording (green line). Greater than 40% respiratory variation in the peak tricuspid E inflow velocity and greater than 25% respiratory variation in the peak mitral E inflow velocity are consistent with constrictive physiology. E_in_ and E_ex_ represent E velocity during inspiration and expiration, respectively.

**Figure 5:** Annulus reversus Tissue Doppler imaging of the medial (A) and lateral (B) mitral annulus. In constrictive pericarditis, tethering of the lateral mitral annulus to the thickened pericardium leads a decrease in diastolic velocity (e’) over the lateral mitral annulus. Concomitantly, the medial e’ progressively increases as the severity of constriction worsens, leading to the characteristic finding of “annulus reversus”.

Following the discovery of his ECP and the terminal nature of his malignancy, the patient wished to defer further procedures and definitive management for the ECP and was discharged to home hospice.

## Discussion

The differential diagnosis for palpitations, dyspnea on exertion, and unintentional weight loss is extensive, and often best approached systematically for comprehensive evaluation. Cardiac etiologies to consider should include ischemia, valvular heart disease, heart failure, restrictive and dilated cardiomyopathies, myocarditis, arrhythmias, conduction disorders, pulmonary hypertension, primary or metastatic malignancy, and pericardial diseases, and to include but not limited to acute pericarditis, constrictive pericarditis, cardiac tamponade, and ECP. There are a plethora of non-cardiac causes, and further evaluation of pulmonary, infectious, gastrointestinal, oncologic, hematologic, and metabolic disorders should all be considered. Anchoring on alternative diagnoses without improvement in clinical condition may lead to deleterious outcomes and delay appropriate treatment. 

The article "Effusive-Constrictive Pericarditis in a Young Active Duty Male" was published in 2020. Journal: Cureus.

This case highlights the unique clinical and pathophysiologic features of ECP along with the importance of comprehensive echocardiography in the evaluation of ECP or other suspected pericardial conditions. With an overall reported prevalence ranging from 1% to 16% in patients presenting with pericarditis or cardiac tamponade, ECP remains a rarely encountered condition [1]. The potential etiologies are diverse and include viral causes, collagen disorders, malignancy, history of radiation, and prior cardiac surgery. In contrast to chronic non-ECP, which predominantly occurs as a post-surgical complication in developed countries, ECP appears to occur more frequently in individuals with a history of radiation or malignancy-related conditions, as was observed in our case [1-7]. Interestingly, our case is unique because it is the first reported case of ECP in a patient with chest wall myoepithelial carcinoma.

While ECP is well described in the literature, it is rarely observed given its low prevalence and complex pathophysiology. Establishing a diagnosis of ECP requires a thorough history and physical examination. In patients presenting with right heart failure, a history of cardiac surgery, tuberculosis, rheumatologic disorders, prior radiation therapy, and/or malignancy should heighten clinical suspicion for constrictive pericarditis, and further evaluation with transthoracic echocardiography should be performed. 

With concomitant features of acute effusive pericarditis, chronic constrictive pericarditis, and in severe cases, cardiac tamponade, identification of ECP by echocardiography requires a comprehensive study with two-dimensional imaging, M-mode, and Doppler echocardiography. Key features of constrictive pericarditis include respirophasic septal shifting, a septal “bounce” or “shudder” due to rapid early diastolic filling of the ventricles, and a plethoric inferior vena cava (IVC) on two-dimensional imaging. Because of lateral wall tethering in CP, “annulus reversus” may also be observed, in which tissue Doppler velocity of the lateral mitral annulus may be abnormally lower than the velocity of the medial mitral annulus [1,2]. In patients with high clinical suspicion, these findings are often sufficient to establish the appropriate diagnosis, thereby reserving invasive hemodynamic evaluation for cases that cannot be established by non-invasive measures.

Once diagnosed, the treatment of ECP should focus on symptomatic improvement and overall quality of life. Initial treatment with diuretic therapy is often considered but is usually minimally effective at palliating symptoms. Historically, the definitive treatment of ECP was limited to pericardiectomy; however, recent studies have shown that ECP may be a transient process that may improve with medication targeted at treating the underlying inflammatory process with either non-steroidal anti-inflammatory agents, corticosteroids, and/or colchicine [1,8]. Despite these findings, optimal medical therapy for ECP remains controversial, and in severe or refractory cases, pericardiectomy may be required for treatment of the condition [1,3].

The article "Effusive-Constrictive Pericarditis in a Young Active Duty Male" was published in 2020. Journal: Cureus.

## Conclusions

ECP is a rare clinical entity demonstrating pathophysiologic properties of constrictive pericarditis in the setting of a persistent pericardial effusion despite treatment with pericardiocentesis. While invasive hemodynamic evaluation by right heart catheterization remains the gold standard in establishing the diagnosis of ECP, non-invasive evaluation with a comprehensive echocardiographic study can often confirm the diagnosis in patients with high pre-test probability. Long-term prognosis of ECP remains unclear; however, with recent studies suggesting that ECP may be a transient condition, conservative treatment should be considered initially, reserving pericardiectomy for severe or refractory cases of ECP. Including ECP on the differential diagnosis of a patient with persistent pericardial effusion can save a patient from extra procedures and result in appropriate treatment sooner.

## References

[1] Kim KH, Miranda WR, Sinak LJ (2018). Effusive-constrictive pericarditis after pericardiocentesis: incidence, associated findings, and natural history. JACC Cardiovasc Imaging.

[2] Klein AL, Abbara S, Agler DA (2013). American Society of Echocardiography clinical recommendations for multimodality cardiovascular imaging of patients with pericardial disease: endorsed by the Society for Cardiovascular Magnetic Resonance and Society of Cardiovascular Computed Tomography. J Am Soc Echocardiogr.

[3] Geske BG, Reddy Y (2019). Pathophysiology and diagnosis of constrictive pericarditis. Am Coll Cardiol.

[4] Oh JK, Welch T (2019). Echocardiography diagnostic criteria for constriction. https://www.acc.org/latest-in-cardiology/articles/2015/03/09/07/22/mayo-clinic-echocardiography-diagnostic-criteria-for-constriction#:~:text=The%20presence%20of%20ventricular%20septal%20shift%20in%20combination%20with%20either,the%20diagnosis%20of%20constrictive%20pericarditis.

[5] Pérez-Casares A, Cesar S, Brunet-Garcia L, Sanchez-de-Toledo J (2017). Echocardiographic evaluation of pericardial effusion and cardiac tamponade. Front Pediatr.

The article "Effusive-Constrictive Pericarditis in a Young Active Duty Male" was published in 2020. Journal: Cureus.

[6] Syed FF, Ntsekhe M, Mayosi BM, Oh JK (2013). Effusive-constrictive pericarditis. Heart Fail Rev.

[7] Jaume S-S, Juan A, Antonio S, Gaietà P-M, Jordi S-S (2004). Effusive-constrictive pericarditis. N Engl J Med.

[8] Feng D, Glockner J, Kim K (2011). Cardiac magnetic resonance imaging pericardial late gadolinium enhancement and elevated inflammatory markers can predict the reversibility of constrictive pericarditis after antiinflammatory medical therapy: a pilot study. Circulation.

